The article "Mechanism of action of Asparagus officinalis extract against multiple myeloma using bioinformatics tools, in silico and in vitro study" was retracted in 2025. Reasons: duplicated images; duplicated data; false authorship; unreliable results or conclusions.

# Mechanism of action of Asparagus officinalis extract against multiple myeloma using bioinformatics tools, *in silico* and *in vitro* study

**DOI:** 10.3389/fphar.2023.1076815

**Published:** 2023-05-09

**Authors:** Yanju Li, Xu Yang, Feiqing Wang, Jianing Zhao, Chike Zhang, Dan Wu, Bo Yang, Rui Gao, Peng Zhao, Yun Zan, Min Su, Zhixu He, Yang Liu, Jishi Wang, Dongxin Tang

**Affiliations:** ^1^ Department of Hematology, Affiliated Hospital of Guizhou Medical University, Guiyang, Guizhou, China; ^2^ Clinical Medical Research Center, The First Affiliated Hospital of Guizhou University of Traditional Chinese Medicine, Guiyang, Guizhou, China; ^3^ Academy of Medical Engineering and Translational Medicine, Tianjin University, Tianjin City, China; ^4^ Key Laboratory of Adult Stem Cell Translational Research, Chinese Academy of Medical Sciences, Guizhou Medical University, Guiyang, Guizhou, China

**Keywords:** multiple myeloma, asparagus, network pharmacology, molecular docking, PI3K/Akt/NF-κB signaling pathway

## Abstract

**Introduction:** Asparagus (*Asparagus officinalis*) is a perennial flowering plant species. Its main components have tumor-prevention, immune system-enhancement, and anti-inflammation effects. Network pharmacology is a powerful approach that is being applied increasingly to research of herbal medicines. Herb identification, study of compound targets, network construction, and network analysis have been used to elucidate how herbal medicines work. However, the interaction of bioactive substances from asparagus with the targets involved in multiple myeloma (MM) has not been elucidated. We explored the mechanism of action of asparagus in MM through network pharmacology and experimental verification.

**Methods:** The active ingredients and corresponding targets of asparagus were acquired from the Traditional Chinese Medicine System Pharmacology database, followed by identification of MM-related target genes using GeneCards and Online Mendelian Inheritance in Man databases, which were matched with the potential targets of asparagus. Potential targets were identified and a target network of traditional Chinese medicine was constructed. The STRING database and Cytoscape were utilized to create protein–protein interaction (PPI) networks and further screening of core targets.

**Results:** The intersection of target genes and core target genes of the phosphoinositide 3-kinase/protein kinase B (PI3K/AKT) pathway was enriched, the top-five core target genes were selected, and the binding affinity of corresponding compounds to the top-five core targets was analyzed using molecular docking. Network pharmacology identified nine active components of asparagus from databases based on oral bioavailability and drug similarity, and predicted 157 potential targets related to asparagus. Enrichment analyses showed that “steroid receptor activity” and the “PI3K/AKT signaling pathway” were the most enriched biological process and signaling pathway, respectively. According to the top-10 core genes and targets of the PPI pathway, AKT1, interleukin (IL)-6, vascular endothelial growth factor (VEGF)A, MYC, and epidermal growth factor receptor (EGFR) were selected for molecular docking. The latter showed that five core targets of the PI3K/AKT signaling pathway could bind to quercetin, among which EGFR, IL-6, and MYC showed strong docking, and the diosgenin ligand could bind to VEGFA. Cell experiments showed that asparagus, through the PI3K/AKT/NF-κB pathway, inhibited the proliferation and migration of MM cells, and caused retardation and apoptosis of MM cells in the G0/G1 phase.

**Discussion:** In this study, the anti-cancer activity of asparagus against MM was demonstrated using network pharmacology, and potential pharmacological mechanisms were inferred using *in vitro* experimental data.

## 1 Introduction

Multiple myeloma (MM) is a hematological malignancy with a worldwide incidence of 160,000 per year and mortality of 106,000 per year (Ludwig et al., 2020). MM is characterized by abnormal clonal plasma cells in the bone marrow, whose uncontrolled growth can lead to devastating bone damage, kidney damage, anemia, and hypercalcemia (Cowan et al., 2022). Despite significant advances in the development of immunomodulatory drugs, proteasome inhibitors, and cluster of differentiation-38-targeting antibodies, 5-year survival of patients is low because of drug resistance and tumor recurrence (Chen et al., 2018). Therefore, safer and more efficacious options are needed urgently.

Traditional Chinese medicine (TCM) is a “treasure” of the Chinese nation. TCM has been used in the clinical adjuvant treatment of many types of malignancies. Studies have shown that use of Chinese herbs alone or as adjuvant therapy can improve tumor-related symptoms, immune function, and quality of life, as well as mitigate adverse effects and prolong survival, in cancer patients (He and Huang, 2020; Zhang et al., 2021).

Asparagus (*Asparagus officinalis*) is a perennial flowering plant species. It has the effect of nourishing Yin and moistening dryness, clearing the lungs, and lowering fire. Asparagus is used to treat all types of wind-dampness and partial paralysis, and to strengthen bone marrow. Asparagus contains saponins, glycosides, flavonoids, phenolic compounds, alkynes, and sulfur-containing compounds (Zhou et al., 2016; Li et al., 2017). The extracts of these compounds have activities against different types of cancer cells, such as inhibition of cell proliferation, induction of apoptosis/cell-cycle arrest, and inhibition of invasion through multiple signaling pathways (Zhang et al., 2020).

Network pharmacology is based on systems biology and multidirectional pharmacology. It can be used to explore the interactions between biological molecules and targets *in vivo* from system-level and biological-network perspectives, thereby enabling effective predictive analysis of drug mechanisms of action, identification of new drug targets (Zhang et al., 2012), and more profound explanation of the mechanisms of interaction between drugs and cells. The mechanisms of action of TCM formulations have yet to be elucidated due to their complex composition and intricate molecules involved in diseases. Molecular docking enables the virtual screening of drugs (Pinzi and Rastelli, 2019). Network pharmacology combined with molecular docking can be used to study the mechanism of action of TCM formulations.

We employed network pharmacology and molecular docking to explore the mechanisms by which asparagus is used to treat MM. The workflow of our study is shown in Supplementary Figure S1.

## 2 Methods and materials

### 2.1 Network pharmacology

#### 2.1.1 Determination of the active ingredients of asparagus

The Traditional Chinese Medicine System Pharmacology (TCMSP) database (www.tcmspw.com/tcmsp.php/) (Ru et al., 2014) was used to ascertain the bioactive components of asparagus. The potential bioactive compounds of ASP were identified according to oral bioavailability (OB) ≥30% and drug-likeness (DL) ≥0.18. The chemical structures of the corresponding compounds were downloaded from the PubChem database (https://pubchem.ncbi.nlm.nih.gov/). The GeneCard database (www.genecards.org/) and Online Mendelian Inheritance in Man (OMIM) database (www.omim.org/) were used to predict and screen of MM targets. R 4.2.1 (R Institute for Statistical Computing, Vienna, Austria) was employed to create Venn diagrams to analyze the intersection of targets between asparagus and MM.

Cytoscape 3.7.2 (www.cytoscape.org/) was used to construct drug compound–disease-target networks and analyze core compounds using the “merge” method. The Search Tool for the Retrieval of Interacting Genes/Proteins (STRING) database ((https://string-db.org/) was used to construct protein–protein (PPI) interaction networks with a confidence of 0.7 and then visualized using. Analyses of enrichment of the function and signaling pathways of genes were done using the Gene Ontology (GO) database (http://geneontology.org/) and Kyoto Encyclopedia of Genes and Genomes (KEGG) database (www.genome.jp/) using R 4.2.1. We prepared a generic target file “drug-disease.txt”, and then ran BioConductor (www.bioconductor.org/) to convert the generic drug-disease target and analyzed the key targets according to the transformed “entrezID”. *p* < 0.05 indicated significant enrichment of genes.

#### 2.1.2 Docking of effective components with key target genes and molecules

The “CytoHubba” plugin was used to analyze PPI networks. Ten core genes were identified: protein kinase B (AKT)1, interleukin (IL)-6, AP-1 transcription factor subunit (JUN), vascular endothelial growth factor (VEGF)A, IL-1B, caspase (CASP)3, hypoxia inducible factor (HIF)-1A, epidermal growth factor receptor (EGFR), matrix metallopeptidase (MMP)-9, and MYC. Analyses of enrichment of signaling pathways showed that the phosphoinositide 3-kinase (PI3K)-AKT signaling pathway was enriched the most. Then, core genes enriched in the PI3K-AKT signaling pathway were selected for molecular docking. The two-dimensional (2D) structures of the core compounds were obtained in the PubChem database. The 3D structures of the core targets were obtained in the Protein Databank (www.rcsb.org/) (Burley et al., 2017), AKT1:3cqu, IL6:1il6, EGFR:5UG9, VEGFA:4kzn, MYC:uniport, 2ovr, predictive structure. PyMol 2.3.4 (https://pymol.org/) was employed to eliminate water molecules, add nonpolar hydrogen to the structure, and save it as a PDBQT file. Autodock Vina 1.1.2 (https://vina.scripps.edu/) was used to dock ligands to target molecules. After molecular docking, the files were visualized through Discovery Studio 2020 (www.3ds.com/). The binding energy was used to evaluate the degree of binding between a molecular compound and its target. The docking results of molecules that exhibited a high degree of binding were visualized using Autodock Vina 1.1.2.

#### 2.1.3 PrognoScan database

The PrognoScan database (http://dna00.bio.kyutech.ac.jp/PrognoScan/) was used to pool all the available datasets and offered a convenient and reliable way to investigate the prognostic values of genes. We used the PrognoScan database to evaluate the prognostic values of core targets molecules across MM. The threshold for included studies for further analysis was set as *p*_corrected_ < 0.05.

### 2.2 Experimental validation

#### 2.2.1 Preparation of asparagus

Pieces of ASP were purchased from GuizhouRen Ji Tang Company Limited (Guiyang, China). First, 50 g of asparagus tablets were weighed. Then, 10-times the volume of water was added, followed by weighing. After soaking for 2 h, extraction was done twice by refluxing (1-h each time). After extraction and filtering, the filtrates were combined. The reduced weight was made-up with water, and the solution concentrated at 70°C under reduced pressure to 1 g/mL of the raw drug. Then, 2 mL of the concentrated solution was removed and diluted to 10 mL with water. The supernatant was filtered through a microporous membrane (0.22 μm). The filtrate was divided into sterile centrifuge tubes and stored at −20°C.

#### 2.2.2 Cell culture

Human MM cell lines (RPMI8226 and U266) were gifts from Professor Jishi Wang (Department of Hematology, Affiliated Hospital of Guizhou Medical University, Guizhou, China). Cells were cultured in RPMI 1640 medium (Gibco, Grand Island, NY, United States) supplemented with 10% fetal bovine serum (BI, Kibbutz, Israel) and 1% penicillin (Solarbio, Beijing, China).

#### 2.2.3 Cell-viability assay

RPMI8226 cells and U266 cells (5 × 104 cells/mL, respectively) were seeded into 96-well plates (100 μL/well) and allowed to incubate overnight at 37°C in a humidified incubator in an atmosphere of 5% CO2. Then, cells were pretreated with asparagus (0, 25, 50, 100, 150, 200, 250 μg/mL) for 1, 2, 3, 4, 5, 6, or 7 days. Next, 20 μL of 3-(4,5-Dimethylthiazol-2-yl)-2,5-diphenyltetrazolium bromide (MTT) solution was added to each well. Then, cells were incubated in an atmosphere of 5% CO_2_ for 4 h at 37°C. Finally, absorbance was measured at 570 nm using a microplate reader (Thermo Fisher Scientific, Waltham, MA, United States). Percent inhibition of cell proliferation was calculated using the following formula:

$$\%\;inhibition\;of\;cell\;proliferation=\left(1-{absorbance}_{experimental\;group}/{absorbance}_{control\;group}\right)\times 100\%$$

#### 2.2.4 Clone formation

Soft agar (1.2 g) was weighed. Three-times the volume of distilled water was added to prepare a 1.2% solution, followed by autoclaving and storage at 4°C. A 20% solution of RPMI 1640 medium was created and set aside. Agarose solution was melted at high temperature and maintained at ∼40°C. The agarose solution was mixed thoroughly (1:1) with the 20% solution of RPMI 1640 medium, and 1 mL added to a five-well plate as an “upper gel” and “lower gel”. Single-cell suspensions containing 2000 RPMI8226 and U266 cells were treated once with to asparagus (0, 50, 100, 200 μg/mL), mixed with soft agar (1:1) as a “middle gel”, placed in an incubator for 21 days, and photographed under a microscope (Nikon, Tokyo, Japan).

#### 2.2.5 5-Ethynyl-2′-deoxyuridine (EdU) assay

RPMI8226 cells and U266 cells in good growth condition were inoculated in six-well plates at 1 × 10^4^ cells/well. Then, RPMI 1640 medium containing 1% fetal bovine serum was added by volume for 12 h to synchronize cells. Then, asparagus (0, 50, 100, 200 μg/mL) was added and incubation allowed for 48 h. After centrifugation (1,000 rpm, 5 min, room temperature), the supernatant was removed, stained with EdU according to manufacturer instructions (RiboBio, Guangzhou, China), and observed and photographed under a fluorescence microscope (Nikon, Tokyo, Japan). The number of EdU-positive cells was calculated using the following formula:

EdU-positive cells (%) = number of red EdU-stained cells/number of blue DAPI-stained cells count × 100.

Where DAPI = 4′,6-Diamidino-2-phenylindole dihydrochloride.

#### 2.2.6 Flow cytometry to measure apoptosis

RPMI8226 cells and U266 cells in good growth condition were inoculated at 1 × 10^5^ cells/bottle in sterile culture flasks (25 cm^2^) and incubated in a CO_2_ thermostat for 12 h. After synchronization, they were treated with asparagus (0, 50, 100, 200 μg/mL) for 48 h. Cells were collected and then centrifuged (1,000 rpm, 5 min, room temperature). After removal of the supernatant, annexin V-fluorescein isothiocyanate (5 μL) and propidium iodide (PI; 5 μL) were added to the cell suspension (500 μL), mixed, and allowed to react for 15 min in the dark at room temperature. Analysis of cells using flow cytometry (BD Biosciences, San Jose, CA, United States) and FlowJo 10.0 software (FlowJo, Ashland, OR, United States).

#### 2.2.7 Flow cytometry to assay the cell cycle

RPMI8226 cells and U266 cells in good growth condition were inoculated at 1 × 10^5^ cells/bottle in sterile culture flasks (25 cm^2^) and incubated in a CO_2_ thermostat for 12 h. After synchronization, cells were replaced with asparagus (0, 50, 100, 200 μg/mL) for 48 h. Cells were collected, washed with pre-cooled phosphate-buffered saline (PBS), centrifuged (2000 rpm, 5 min, room temperature) and resuspended in pre-cooled PBS. The cell suspension was added to precooled 70% ethanol and fixed overnight at 4°C. The supernatant was washed twice with PBS, then PI (450 μL) and RNase A (50 μL) were added and incubation allowed for 30 min at 4°C. Finally, the cell cycle was evaluated by flow cytometry and data analyzed using FlowJo 10.0 (www.flowjo.com/).

#### 2.2.8 Cell invasion

The migration and invasion capacities of cells were determined using the Transwell™ assay (Corning, Corning, NY, United States). To test the migration ability of RPMI8226 and U266 cells, 1 × 10^5^ cells (200 μL) were placed in the upper compartment of a Transwell chamber (8 µm) and asparagus (0, 50, 100, 200 μg/mL) added according to experimental requirements. Then, RPMI 1640 medium containing 20% fetal bovine serum (600 μL) was added to the lower compartment. After 48 h, cells in the upper compartment were wiped off. Next, 10 μL of MTT (10 mg/mL) was added to each well and incubation allowed for 4 h at 37°C. The supernatant was removed, dimethyl sulfoxide (150 μL) was added, and the reaction allowed to proceed for 15–20 min. The absorbance at 570 nm was measured using an automatic microplate reader (Thermo Fisher Scientific, Waltham, MA, United States).

#### 2.2.9 Immunofluorescence staining

RPMI8226 and U266 cells after 48 h treatment with asparagus (0, 50, 100, 200 μg/mL) were fixed, punched, and incubated overnight with primary antibody (nuclear factor-kappa B (NF-κB), dilution = 1:100). Subsequently, cells were incubated with fluorescent secondary antibody (goat anti-rabbit IgG, dilution = 1:100) for 1 h in the dark at room temperature. Finally, DAPI was added. An inverted fluorescence microscope was used to observe cells and acquire images. All experiments are repeated three times.

#### 2.2.10 Western blotting

After RPMI8226 and U266 cells were treated with asparagus (0, 50, 100, 200 μg/mL) for 48 h, the cells were collected for protein extraction. Extraction of total protein from cells/tissues containing protease inhibitors, phosphatase inhibitors, and PMSF (Solarbio, Beijing, China) by radioimmunoprecipitation (RIPA) lysis buffer. Equal amounts of protein were separated by sodium dodecyl sulfate–polyacrylamide gel electrophoresis (Solarbio, Beijing, China) using 6%–12% gels and then transferred to polyvinylidene fluoride (PVDF) membranes (0.45 µM; Millipore, Bedford, MA, United States). Next, 5% skimmed milk was employed to block PVDF membranes for 1 h at room temperature. PVDF membranes were probed with the primary antibodies (at 1:1,000 dilution) Bax, B-cell lymphoma (Bcl)-2, β-actin, P21, NF-κB, PI3K, phosphorylated (P)-PI3K, AKT, P-AKT (all from Beyotime Institute of Biotechnology, Shanghai, China), C-myc, cyclin D1 (CCND1), SRY-box 2 (SOX2), Homeobox protein NANOG (NANOG), octamer-binding transcription factor (OCT)4 (all from Proteintech), and N-cadherin (Cell Signaling Technology, Danvers, MA, United States). Then, PVDF membranes were probed with goat anti-rabbit and goat anti-mouse horseradish peroxidase-coupled secondary antibodies (1:5,000 dilution; Boster Biotechnology, Wuhan, China). PVDF membranes were incubated gently overnight at 4°C. The next day, PVDF membranes were rinsed thrice with Tri-buffered saline-Tween 20 (Solarbio) and incubated with goat anti-rabbit or goat anti-mouse horseradish peroxidase-conjugated secondary antibodies for 2 h at room temperature. Finally, an ultra-sensitive electrochemiluminescence reagent was used with substrates (Boster Biotechnology) on the immune-responsive protein bands. ImageJ (US National Institutes of Health, Bethesda, MD, United States) was employed to quantify protein bands according to gray values normalized to the β-actin level. All experiments are repeated three times.

### 2.3 Statistical analyses

Statistical evaluations were undertaken using Prism 8.3.1 (GraphPad, San Diego, CA, United States). Data are the mean ± SD. Results were evaluated using one-way analysis of variance. *p* < 0.05 was considered significant.

## 3 Results

### 3.1 Active ingredients of asparagus

Based on the screening criteria of OB ≥ 30% and DL ≥ 0.18, nine active ingredients of asparagus were retrieved from the TCMSP database (Table 1). These nine active ingredients corresponded to 172 targets (Supplementary Table S1).

**TABLE 1:** Activate compounds of asparagus according to the TCMSP database.

Mol ID	Molecule name	Pubchem CID	OB (%)	DL
MOL000358	beta-sitosterol	222,284	36.91	0.75
MOL000359	sitosterol	12,303,645	36.91	0.75
MOL003889	methylprotodioscin_qt	1,62,818,391	35.12	0.86
MOL003891	pseudoprotodioscin_qt	10,573,853	37.93	0.87
MOL003896	7-Methoxy-2-methyl isoflavone	354,368	42.56	0.2
MOL003901	Asparaside A_qt	No	30.6	0.86
MOL000449	Stigmasterol	5,280,794	43.83	0.76
MOL000546	Diosgenin	99,474	80.88	0.81
MOL000098	Quercetin	5,280,343	46.43	0.28

### 3.2 PPI networks

A total of 277 related genes were screened from seven compounds: beta-sitosterol, sitosterol, pseudoprotodioscin_qt, 7-Methoxy-2-methyl isoflavone, stigmasterol, diosgenin, and quercetin. A total of 3,510 targets related to MM treatment were obtained from GeneCard and OMIM databases. We used R 4.2.1 to input potential targets screened by MM and targets acted upon by the active component of asparagus, and yielded 125 intersecting genes (Figure 1A). The “drug-active compaction-target” network diagram constructed by Cytoscape 3.7.2 reflected the correspondence of compound targets (Figure 1B). The 125 predicted cross-targets of asparagus and MM were imported into the STRING database, and the selected species were *Homo sapiens* with a confidence level >0.7. Diagrams to represent PPI networks were generated to obtain protein-interaction relationships (Figure 1C). Cross-targets were imported into Cytoscape 3.7.2 to create a network diagram of potential target interactions (Figure 1D). Nodes represented proteins and edges represented relationships between proteins. The degree value was represented by colors from red to yellow, and from large to small. According to the top-20 core genes of the degree value (Figure 1E), the PPI network was analyzed by the Cytohubba plug-in and, finally, 10 core genes were obtained: AKT1, IL-6, VEGFA, IL-1B, CASP-3, C-X-C motif chemokine ligand (CXCL)-8, EGFR, MMP-9, and MYC (Figure 1F).

**FIGURE 1:** Diagram showing a drug–active ingredient–target network and Venn diagram. **(A)** Venn diagram, blue represents the MM target, pink represents the asparagus target, and shaded areas represent the asparagus and MM crossover targets. **(B)** Diagram showing a drug–active ingredient–target network. **(C)** Target proteins interaction network. In this network, nodes represent proteins, lines represent functional associations between proteins, and the line thickness corresponds to the confidence level of the reported association. **(D)** The PPI network was constructed using a search tool to retrieve plug-in targets from a database of interacting genes/proteins that were imported into Cytoscape, where the targets are candidates for use in MM therapy. Proteins are indicated by nodes on the right (colors from red to purple indicate the degree of medicinal-target interactions). Edges indicate protein–protein associations. **(E)** Histogram showing the protein-interaction relationship of MM. **(F)** Top-10 targets (central targets) in the PPI network ranked by maximum group centrality using the “cytoHubba” plug-in.

### 3.3 Enrichment analyses using GO and KEGG databases

We wished to further explore the possible mechanism of action of 125 candidate targets for MM treatment. Enrichment analyses of candidate targets were done based on GO and KEGG databases using R 4.2.1.

According to the GO database, key proteins regulated 137 biological processes, mainly “DNA-binding transcription factor binding”, “steroid hormone receptor activity”, “cytokine receptor binding”, and “transcription coactivator”. Values for binding energy showed the top-20 biological processes (Figure 2A). Analyses of enrichment of signaling pathways using the KEGG database revealed 138 terms. The top-20 signaling pathways were screened for MM-related pathways based on *p*_adjusted_ < 0.05 (Figure 2B). Among them, the most important signaling pathways were “mitogen-activated protein kinase” (MAPK), HIF-1, PI3K-AKT, tumor necrosis factor, and other pathways related to immunity and inflammation. The PI3K/AKT/NF-κB signaling pathway was the most enriched. PI3K/AKT/NF-κB signaling pathway-related target maps are shown as Figure 2C. Target genes in the PI3K/AKT signaling pathway are shown in Table 2. Asparagus may regulate the proliferation and apoptosis of cells through the PI3K/AKT signaling pathway for MM treatment. Therefore, we selected the PI3K/AKT/NF-κB pathway for further exploration to identify potential mechanisms by which asparagus affects MM.

**FIGURE 2:** Enrichment analyses of function and signaling pathways using the Gene Ontology database and Kyoto Encyclopedia of Genes and Genomes database. **(A)** The larger the bar (left), the higher is the level of enrichment for each biological process, and the color of the bar represents the level of gene enrichment for each biological process. The names of biological processes, cellular components, and molecular functions are distributed in the vertical coordinate and the degree of enrichment in the horizontal coordinate. Air bubble diagram (right) the size of the points represents the number of genes; the larger the point, the higher the number of genes in the corresponding process. **(B)** Air bubble diagram (right) the size of the points represents the number of genes; the larger the point, the higher the number of genes in the corresponding process (left) names of pathways distributed in vertical coordinates and the number of genes enriched in the pathways distributed in horizontal coordinates. *p*-values indicate the importance of enrichment; the lower the *p*-value, the redder the color of the graph, the higher the enrichment. **(C)** PI3K/AKT/NF-κB pathway for treatment of MM using asparagus, with the target genes of asparagus marked in red.

**TABLE 2:** Target genes in the PI3K/AKT pathway.

Passage name	Name of target genes on the pathway
PI3K/AKT	GSK3B, CDKN1A, RELA, EGFR, CASP9, RXRA, ERBB3, CCND1, MYC, ERBB2, SPP1, AKT1, MAPK1, CHUK, EGF, NOS3, INSR, IGF2, PRKCA, IL2, MTOR, VEGFA, COL1A1, IL6, BCL2, RAF1, BCL2L1

### 3.4 Verification by molecular docking

Molecular docking was used to verify the binding ability of two active ingredients of asparagus, iosgenin and quercetin, to key genes, which were selected from the intersection of the top-10 core genes of PPI networks and genes identified in the PI3K/AKT pathway (AKT1, VEGFA, IL-6, EGFR, MYC) (Table 3). Binding energy was used to evaluate the degree of docking, and binding energy ≤ −5 kcal/mol denoted that binding could occur, and ≤ −7 kcal/mol indicated good binding ability (Li et al., 2019).

**TABLE 3:** Bioactive compounds with targets.

Molecular ID	Compounds	Candidate targets
MOL000546	diosgenin	AKT1, VEGFA
MOL000098	quercetin	AKT1, VEGFA, IL-6, NFKB1A, EGFR, MYC

Diosgenin targeted the AKT1 residues GLU-228, TYRA-176, and THRA-172 by hydrogen bonding (Figure 3). AKT1 bound weakly to diosgenin (docking fraction = −2.2 kcal/mol) (Supplementary Table S2). VEGFA interacted with the residue GLNA-87 by linking diosgenin to hydrogen bonds (Figure 3) with a docking fraction of −6.6 kcal/mol. Based on a docking fraction = −4.6 kcal/mol, quercetin bound weakly to the AKT1 residues AGLUA-228 and ARGA-174 (Figure 3). IL-6 interacted strongly with quercetin (docking fraction = −7.2 kcal/mol), as well as ARGA-169, and ASNA-62 targeted to quercetin *via* hydrogen bonding (Figure 3). EGFR interacted with quercetin (Figure 3) by hydrogen bonding to two residues of quercetin (THRA-243 and VALA-39) with a docking fraction of −7.7 kcal/mol. Based on a docking fraction of −5.1 kcal/mol, quercetin was targeted to VEGFA *via* hydrogen bonding of ARGA-82 (Figure 3). Quercetin was targeted to MYC by binding hydrogen bonds to TRPB-2425, ARGB-2505, METB-287, LEUB-2547 and nobiletin based on a docking fraction of −8.4 kcal/mol (Figure 3).

**FIGURE 3:** **(A)** Chemical structures of quercetin and nobiletin. **(B)** Tertiary structure of the proteins AKT1, EGFR, IL-6, VEGFA, and MYC. **(C)** Molecular-docking model for major compounds.

### 3.5 Prognostic value of five target genes in MM

Associations between five target genes (AKT1, EGFR, IL-6, MYC, VEGFA) and the survival outcomes of MM patients based on the overall survival (OS) were determined using the PrognScan database (Mizuno et al., 2009). Lower expression of EGFR was associated with a poor prognosis in MM patients. Aberrant regulation of AKT1, MYC, and VEGFA may contribute to the tumorigenesis and development of MM (Figure 4). However, only VEGFA expression was significant in terms of the prognosis of MM patients.

**FIGURE 4:** **(A)** Kaplan–Meier survival curves comparing samples with high expression of five molecules with those with low expression in MM datasets using a Kaplan–Meier plotter.

### 3.6 Asparagus inhibited the proliferation of MM cells *in vitro*

MM cells (RPMI8226 and U266) were pretreated with asparagus (0, 50, 100, 200 μg/mL) from 1 day to 7 days (Figure 5A). The median inhibitory concentrations of RPMI8226 cells and U266 cells were 209.4 ug/mL and 162.39 ug/mL at 48 h and 164.7 ug/mL and 107.6 ug/mL at 72 h, respectively (Figure 5B). Light microscopy showed that, with an increase in the asparagus concentration, the number of cells decreased gradually; cells shrank, and different degrees of nuclear consolidation/vacuolation occurred (Figure 5C).

**FIGURE 5:** Asparagus inhibited the proliferation of RPMI8226 cells and U266 cells. **(A)** MTT assay of MM cell lines (RPMI8226 and U266 cells) after 1–7 days of treatment with indicated doses of asparagus. **(B)** Median inhibitory concentration (IC_50_) of asparagus in RPMI8226 cells and U266 cells at 48 h. **(C)** Morphological changes in cells were observed under a light microscope after 48 h of treatment with asparagus.

We used clone-formation experiments and the EdU assay to study the effect of asparagus on the proliferation of MM cells (RPMI8226 and U266). After 21 days, cell-clone formation was reduced significantly after asparagus addition compared with that in the control group (Figure 6A). The EdU assay showed that cell proliferation was reduced significantly after asparagus addition compared with that in the control group (Figure 6B). These results suggested that asparagus inhibited the viability of MM cells.

**FIGURE 6:** **(A)** Changes in cell morphology after action of asparagus on MM cells for 48 h (×10 magnification). **(B)** Clone formation after action of asparagus on MM cells for 21 days (×10 magnification). **(C)** Statistics of clone formation. **(D)** EdU assay to measure cell proliferation for 48 h (×10 magnification). (^*^ *p* < 0.05, ^**^ *p* < 0.01, ^***^ *p* < 0.001, ^****^ *p* < 0.0001).

We wished to determine the ability of asparagus to induce cell-cycle arrest. Flow cytometry was employed to study the number of MM cells in each phase of the cell cycle. As the asparagus concentration increased, the number of cells in G1 phase was significantly higher than that in the control group (Figure 7A), and the number of cells in the S phase decreased. In addition, we used protein blotting to measure changes in expression of relevant proteins after treating MM cells with asparagus for 48 h. Expression of c-Myc and CCND1 was downregulated significantly, and p21 expression was upregulated significantly, with increasing asparagus concentration (Figure 7B). These data suggested that asparagus induced cell-cycle arrest in the G1 phase, thereby affecting the proliferation of MM cells.

**FIGURE 7:** **(A)** Flow cytometry of MM cells 48 h after asparagus treatment (n = 3 per group). **(B)** Expression of cyclin D1 after treatment of MM cells with asparagus (n = 3 per group). (^*^ *p* < 0.05, ^**^ *p* < 0.01, ^***^ *p* < 0.001).

### 3.7 Asparagus induces the apoptosis of MM cells

We investigated the effect of asparagus on the apoptosis of MM cells by flow cytometry. Percent apoptosis was significantly higher in RPMI8226 cells and U266 cells with increasing asparagus concentrations compared with that in the control group (Figure 8A). We wished to investigate the molecular mechanism of apoptosis in asparagus-treated MM cells. We measured expression of apoptosis-related proteins in MM cells treated with asparagus for 48 h by protein blotting (Figure 8B). With an increase in the asparagus concentration, Bcl-2 expression in MM cells was lower, and Bax expression was significantly higher, than that of the control group. These data suggested that asparagus could induce the apoptosis of MM cells.

**FIGURE 8:** **(A)** Flow cytometry showing apoptosis of MM cells after asparagus treatment of MM cells (n = 3 per group). **(B)** Western blots of apoptotic proteins after asparagus treatment of MM cells (n = 3 per group). (^*^ *p* < 0.05, ^**^ *p* < 0.01, ^***^ *p* < 0.001).

### 3.8 Asparagus inhibits invasion by MM cells

We investigated the effect of asparagus on the invasion ability of MM cells (RPMI8226 and U266) (Figure 9A). Compared with the control group, the invasion ability of RPMI8226 cells and U266 cells was reduced significantly (*p* < 0.05) after addition of asparagus (50, 100, 200 μg/mL), and the difference was concentration-dependent. Protein expression of N-cadherin in RPMI8226 cells and U266 cells was reduced significantly with increasing asparagus concentration, whereas protein expression of E-cadherin was increased significantly (Figure 9B). Hence, asparagus inhibited invasion by MM cells.

**FIGURE 9:** **(A)** Absorbance values showing migration of MM cells 48 h after asparagus treatment. **(B)** Expression of related migratory proteins 48 h after asparagus treatment (n = 3 per group). **(C)** Statistical analyses of related proteins. (^*^ *p* < 0.05, ^**^ *p* < 0.01, ^***^ *p* < 0.001).

### 3.9 Asparagus regulates the “stemness” of MM cells

Protein blotting showed that expression of the stemness-related genes Nanog, SOX2, and OCT4 was reduced significantly in MM cells under the influence of asparagus. These results suggested that asparagus may reduce the stemness of MM cells (Figure 10).

**FIGURE 10:** Protein expression of related stemness factors (OCT4, SOX2, NANOG) in RPMI8226 cells and U266 cells after treatment with asparagus (50, 100, 200 μg/mL). (^*^ *p* < 0.05, ^**^ *p* < 0.01, ^***^ *p* < 0.001, ^****^ *p* < 0.0001).

### 3.10 Effect of asparagus on the PI3K/AKT/NF-κB signaling pathway

We analyzed NF-κB localization by the immunofluorescence assay. Blue fluorescence by DAPI staining denoted the nucleus and red fluorescence indicated NF-κB, compared with the control group. NF-κB translocated from inside to outside the nucleus after asparagus (200 μg/mL) treatment (Figure 11A). We analyzed the effect of asparagus on the PI3K/AKT/NF-κB pathway in MM cells. Western blotting showed that protein expression of p-PI3K, p-AKT, and NF-κB decreased significantly with increasing asparagus concentration, whereas protein expression of PI3K and AKT did not change significantly (Figure 11B). These findings suggested that the PI3K/AKT/NF-κB pathway was involved in the induction of apoptosis of MM cells after asparagus treatment.

**FIGURE 11:** **(A)** NF-κB localization using an immunofluorescence assay (10×). **(B)** PI3K/AKT/NF-κB pathway-related protein expression (n = 3 per group). (^*^ *p* < 0.05, ^**^ *p* < 0.01, ^***^ *p* < 0.001, ^****^ *p* < 0.0001).

## 4 Discussion

A lack of scientific evidence and clear molecular mechanisms and targets have hindered TCM development worldwide (Wang et al., 2018). Network pharmacology is a powerful approach that is being applied increasingly to research of herbal medicines. Herb identification, study of compound targets, network construction, and network analysis have been used to elucidate how herbal medicines work. We applied network pharmacology to investigate the regulatory mechanism of an aqueous extract of asparagus in MM cells. We conducted *in vitro* experiments to validate these results to elucidate the mechanism of action of asparagus in MM treatment.

Numerous studies have shown that asparagus has exert anti-tumor activity by targeting multiple signaling and metabolic pathways *in vitro* and *in vivo* (Cheng et al., 2021; Xu et al., 2021; Liang et al., 2022). Asparagus contains steroidal saponins, glycans, flavonoids, phenolic compounds, alkynes, and sulfur-containing compounds. These extracted compounds can inhibit tumor-cell proliferation, block the cell cycle to induce apoptosis, and show similar inhibitory effects on different types of tumor cells (Wang et al., 2013; Zhang et al., 2020). We showed that an aqueous extract of asparagus could improve anticancer effects substantially by apoptosis induction. Flow cytometry indicated that an aqueous extract of asparagus induced marked apoptosis of MM cells compared with that in the control group.

Apoptosis is associated with various biological processes linked to tumorigenesis. Flow cytometry indicated that asparagus induced the apoptosis of MM cells. Immunoblotting revealed that asparagus upregulated expression of the pro-apoptotic protein Bax and downregulated expression of the anti-apoptotic protein Bcl-2. The Bax/Bcl-2 ratio is crucial for determining the entry of cells into the apoptotic pathway (Ramesh and Medema, 2020). Thus, our data suggest that asparagus induces the apoptosis of MM cells through internal regulation of several key proteins.

Clone-formation experiments revealed that asparagus inhibited the proliferation of MM cells in a dose-dependent manner. Also, asparagus induced cycle arrest of MM cells in the G1 phase. Aberrant regulation of the cell cycle has been shown to be associated with the genesis and progression of tumor cells. Unregulated growth is a unique feature of cancer cells, but also a major requirement in carcinogenesis (Lu et al., 2005). Cell proliferation is controlled by cytoplasmic proteins involved in the cell cycle (Vermeulen et al., 2003). Therefore, we selected target genes downstream of the PI3K/AKT/NF-κB pathway related to the cell cycle based on the KEGG database, and measured expression of cell cycle-related proteins. Protein blotting showed that treatment with asparagus resulted in downregulation of expression of CCND1 and c-Myc, and upregulation of p21 expression. CCND1 positively regulates the cell cycle, and its overexpression shortens the G1 phase of cells. These actions lead to excessive cell proliferation and promote the genesis and progression of tumors. p21 is an inhibitor of cell cycle protein-dependent kinase and plays an important part in controlling cell-cycle progression (Hartwell and Kastan, 1994). c-Myc is an important gene that marks the proliferative state of cells (Elbadawy et al., 2019). p21 expression has been found to be associated with expression of CCND1 and c-Myc. p21 inhibits DNA replication by interacting with c-Myc, leading to cell-cycle arrest in the G1 phase (Claassen and Hann, 2000). Taken together, these results suggest that asparagus can inhibit the proliferation of MM cells by reducing expression of CCND1 and c-Myc and increasing p21 expression, to block MM cells from the G1 phase to S phase.

The PI3K/AKT signaling pathway is an important player in MM genesis. It is closely associated with the proliferation and migration of MM cells, angiogenesis, and drug resistance (Tai et al., 2003; Liu et al., 2020a; Peng et al., 2020; He et al., 2021). The PI3K/AKT pathway has emerged as a promising therapeutic strategy against MM (Mimura et al., 2014). We measured expression of proteins in the PI3K/AKT/NF-κB pathway using protein blotting. Asparagus inhibited expression of P-PI3K, P-AKT1, and NF-κB in a dose-dependent manner. The immunofluorescence assay showed that asparagus inhibited the entry of NF-κB into the nucleus. We hypothesize that asparagus may inhibit the malignant features of MM cells by blocking the PI3K/AKT/NF-κB signaling pathway. AKT has a key regulatory role in MM pathophysiology (including survival, proliferation, and metabolism) and has emerged as a key therapeutic target (Song et al., 2018). VEGF is a core pro-angiogenic cytokine and is associated with disease progression in MM patients. Studies have shown that increased expression of AKT and PI3K promotes the proliferation of MM cells (U266 and RPMI-8226), yet VEGF increases angiogenesis and promotes MM growth (Liu et al., 2020b).

It has been shown that the PI3K/Akt/NF-κB signaling pathway is involved in epithelial–mesenchymal–transition (EMT) and cell invasion. We found that inhibition of the PI3K/AKT/NF-κB signaling pathway by asparagus led to the invasion ability of MM cells to decrease. Asparagus treatment increased expression of E-cadherin and reduced expression of N-cadherin, which are EMT markers in RPMI8226 and U266 cells. These results suggest that asparagus can inhibit EMT in MM cells. EMT is also a significant factor in the metastasis of MM cells (Peng et al., 2020; Babaei et al., 2021).

Despite tremendous advances in MM treatment, the 5-year survival of patients is ∼47%. This poor survival is due mainly to drug resistance and tumor relapse. The stem cell-associated transcription factors NANOG, OCT4, and SOX2 are associated with drug resistance and relapse in MM patients (Wang et al., 2022). We measured expression of NANOG, OCT4, and SOX2 in RPMI8226 cells and U266 cells by protein immunoblotting. We found that asparagus inhibited expression of NANOG, OCT4, and SOX2 in MM stem cells, thereby suggesting that asparagus could be a new therapeutic target for reversing chemoresistance in patients with refractory/relapsed MM.

## 5 Conclusion

We explored the pharmacological mechanism of action of asparagus on MM. Asparagus exerted antitumor activities (proliferation inhibition, cell-cycle arrest, induction of apoptosis, reduction of invasion) of MM cells. Asparagus may exert its anti-MM effects by inhibiting the PI3K/AKT/NF-κB signaling pathway. Our study provides a theoretical and experimental basis for the application of asparagus as an antitumor agent.

## Data Availability

The original contributions presented in the study are included in the article/Supplementary Materials, further inquiries can be directed to the corresponding author.
